The article "Millennium Development Goals 4 and 5: progress and challenges" was published in 2013. Journal: BMC Med.

# Millennium Development Goals 4 and 5: progress and challenges

**DOI:** 10.1186/1741-7015-11-225

**Published:** 2013-10-16

**Authors:** Jennifer Bryce, Robert E Black, Cesar G Victora

**Affiliations:** 1 Institute for International Programs, Johns Hopkins Bloomberg School of Public Health, 615 N Wolfe Street, Baltimore, MD 21205, USA; 2 Postgraduate Program in Epidemiology, Federal University of Pelotas, Pelotas, Brazil

**Keywords:** Child survival, Child mortality, Maternal survival, Maternal health, Maternal mortality, Neonatal mortality, Nutrition, Millennium Development Goals

## Abstract

The Millennium Development Goals have galvanized efforts to improve child survival (MDG-4) and maternal health (MDG-5). There has been important progress on both MDGs at global level, although it now appears that few countries will reach them by the target date of 2015. There are known and efficacious interventions to address most of the major causes of these deaths, but important gaps remain. The biggest challenge is to ensure that all women and children have access to life-saving interventions. Current levels of intervention coverage are too low, representing missed opportunities. Providing services at the community level is an important emerging priority, but preventing maternal and neonatal deaths also requires access to health facilities. Readers of the *Medicine for Global Health* collection^a^ in *BMC Medicine* are urged to make maternal and child health one of their key concerns, even if they work on other topics.

## Background

The eight Millennium Development Goals (MDGs) arose out of the United Nations Millennium Declaration of 2000, and set targets for levels of achievement for the period from 1990 to 2015 [1]. MDG-4, ?Reduce child mortality?, has a target of reducing the under-five mortality rate by two-thirds. MDG-5, ?Improve maternal health?, has a target of reducing the maternal mortality ratio by three-quarters. Despite important limitations [2], the MDGs have galvanized and focused global attention and monitoring. MDGs 4 and 5 are important for global health as a whole, because they represent the mortality endpoints for women and children across specific diseases, nutritional and environmental risk factors, and more distal determinants including inequalities in economic resources and education. Under-five mortality is also one of the major determinants of life expectancy across the globe. In this brief commentary, we review progress regarding MDG-4 and MDG-5 in the 75 low- and middle-income countries (LMIC) that account for over 95% of maternal and child deaths [3].

### The changing epidemiology of women?s and children?s health

Progress on MDG-4 for child survival has been impressive at the global level, although it now appears clear that the global target will not be reached [4]. The number of deaths among children under five worldwide has decreased from 12.4 million [1] in 1990 to 7.6 million in 2010 [5], a reduction of nearly 40% in spite of an increase in the number of births. Child deaths continue to be concentrated in LMICs, and increasingly in sub-Saharan Africa and South Asia [5]. Pneumonia, diarrhea and malaria together accounted for over 30% of under-five deaths in 2010, with three-quarters of deaths due to major infections occurring in the first two years of life [6]. Under-nutrition contributes to nearly half of all child deaths [7]. As deaths in the 1- to 59-month age group decline, deaths in the first 28 days (neonatal deaths) represent a growing proportion of all under-five deaths. The major causes of neonatal deaths in 2010 were preterm birth complications, intrapartum complications and pneumonia/sepsis [5].

Progress on MDG-5 for maternal health has been slower than for MDG-4, with deaths declining from around 400,000 to around 275,000 [8,9]. The major causes of maternal deaths in 2010 are estimated to have been hemorrhage (22.9%), hypertensive disorders (18.5%), abortion (14.6%), sepsis (8.6%), and other direct and indirect causes (35.5%) [10].

### What interventions are available, and where are the gaps?

There has been important progress in identifying interventions to reduce mortality from the major causes of child deaths, but gaps remain. For pneumonia, the newly-implemented vaccine for pneumococcal disease holds potential for sizable impact, but fails to protect against prevalent serotypes in some LMICs [11]. Antibiotic treatment of bacterial pneumonia is highly efficacious, but may be compromised by increasing resistance of bacteria to inexpensive antibiotics [12]. There is no available treatment or vaccines for important viral causes of lower respiratory illness, such as Respiratory Syncytial Virus. For diarrhea, rotavirus is the most important cause of severe childhood diarrhea globally, but the vaccine that is currently implemented appears to provide only about 50% protection in low-income countries [6]. Oral rehydration salts (ORS) solution and zinc are effective treatments, but coverage remains too low [3]. For malaria, early results suggest that the currently available vaccine may offer only modest protection of young children in highly endemic areas [13,14]. Long-lasting insecticide-treated nets that extend the period of protection from 6 to 12 months to three years or longer have been scaled up in the majority of countries where *Plasmodium falciparum* is a major cause of child deaths, but the duration of protection varies by product and remains under investigation [15,16]. Moreover, resistance to anti-malarial drugs is emerging [13,17]. One important advance is the development and scaling up of rapid diagnostic tests to allow better targeting of treatment for both malaria and pneumonia.

Preventing neonatal and maternal deaths is challenging, especially where access to health facilities is limited. Chlorhexidine, which is an antiseptic and disinfectant agent, applied to the umbilical cord at birth reduces deaths related to neonatal infection and is ready for implementation [18]. However, preventing intrapartum complications, such as obstructed labor and hemorrhage, two leading causes of maternal deaths, managing babies that are born very early, and treating neonatal sepsis, all require good practices at the time of labor and delivery and preferably access to health facilities.

### Achieving and sustaining high and equitable coverage

The real challenge in preventing unnecessary deaths among women and children is ensuring that high-impact interventions are available on demand and used by every woman and child who needs them. Figure?1 shows the latest available median coverage rates for a selection of interventions and service contacts across the continuum of care from reproductive through maternal, neonatal and child health tracked by Countdown to 2015 for Maternal, Newborn and Child Survival [3]. With the exception of vaccines and vitamin A supplementation, all interventions are being severely under-utilized. Coverage is high for some service contacts (for example, antenatal care), but little is known about whether these opportunities to deliver interventions are actually being used [19]. New strategies for delivering interventions at the community level and ensuring the continuous availability of essential commodities are being adopted and implemented by countries, but not fast enough. Within-country inequalities are also important. In virtually every Countdown country, coverage tends to be lower among the poorest families.

**Figure 1:** **Intervention coverage and service contacts along the continuum of care.** Median national coverage of interventions in Countdown countries based on the most recent measurement since 2006 (%). Source: Adapted from Countdown to 2015 for Maternal, Newborn and Child Survival, 2012.

The reasons why few Governments in low-income countries have been able to achieve high, sustained and equitable coverage for interventions proven to reduce maternal and child deaths vary by setting and are not fully understood. Certainly resources - both foreign aid and domestic investments - are a limiting factor [20,21], as are competing global priorities that do not always focus on the major causes of death. Rapid gains in coverage for insecticide-treated nets for malaria prevention and complex interventions to reduce maternal-to-child transmission of HIV demonstrate what can be done given adequate political will and external financing [22]. Conflict and limited technical capacity at country level are also important impediments. However, the interplay of these factors at national and sub-national levels in the highest-burden countries needs further research, and there is unlikely to be a ?one-size-fits-all? solution.

### Future directions and conclusions

The MDGs have focused efforts on reduction of maternal and child mortality. In the post-2015 era, the health of women and children must remain a priority, and the MDG targets must be extended. Governments must be empowered to address the major causes of mortality in their context, but the lens should be expanded to include maternal morbidity, maternal and child nutrition, and child development. Programs must have the capacity to identify the women and children who are not being reached, and to develop local solutions for ensuring that even those disenfranchised by poverty, ethnicity, gender or conflict have continuous access to services delivered at levels of quality that ensure their effectiveness [23]. Researchers and practitioners, including all those who follow the *Medicine for Global Health* collection, must ensure that the health of women and children in LMICs is properly addressed, whatever the specific focus of their research. The biggest challenge ahead is to combat complacency, and to recognize that the gains made to date only increase our responsibility to ensure that no woman, mother, baby or child dies unnecessarily.

## Endnote

^a^Please see the Medicine for Global Health article collection: http://www.biomedcentral.com/bmcmed/series/MGH.

## Abbreviations

LMIC: Low- and middle-income country; MDG: Millennium Development Goal; ORS: Oral rehydration salts.

## Competing interests

The authors declare that they have no competing interests.

## Authors? contributions

JB prepared the outline, which was reviewed and approved by all the authors. JB and RB prepared the first draft. All authors contributed to subsequent drafts, and read and approved the final manuscript.
